# Nanoparticles: A Potential and Effective Method to Control Insect-Borne Diseases

**DOI:** 10.1155/2023/5898160

**Published:** 2023-05-11

**Authors:** Danyue Nie, Jiaqiao Li, Qinghua Xie, Lele Ai, Changqiang Zhu, Yifan Wu, Qiyuan Gui, Lingling Zhang, Weilong Tan

**Affiliations:** ^1^Nanjing Bioengineering (Gene) Technology Center for Medicines, Nanjing 210002, China; ^2^Fujian Agriculture and Forestry University, Fuzhou 350002, China

## Abstract

Insects act as vectors to carry a wide range of bacteria and viruses that can cause multiple vector-borne diseases in humans. Diseases such as dengue fever, epidemic encephalitis B, and epidemic typhus, which pose serious risks to humans, can be transmitted by insects. Due to the absence of effective vaccines for most arbovirus, insect control was the main strategy for vector-borne diseases control. However, the rise of drug resistance in the vectors brings a great challenge to the prevention and control of vector-borne diseases. Therefore, finding an eco-friendly method for vector control is essential to combat vector-borne diseases. Nanomaterials with the ability to resist insects and deliver drugs offer new opportunities to increase agent efficacy compared with traditional agents, and the application of nanoagents has expanded the field of vector-borne disease control. Up to now, the reviews of nanomaterials mainly focus on biomedicines, and the control of insect-borne diseases has always been a neglected field. In this study, we analyzed 425 works of the literature about different nanoparticles applied on vectors in PubMed around keywords, such as“nanoparticles against insect,” “NPs against insect,” and “metal nanoparticles against insect.” Through these articles, we focus on the application and development of nanoparticles (NPs) for vector control, discussing the lethal mechanism of NPs to vectors, which can explore the prospect of applying nanotechnology in the prevention and control of vectors.

## 1. Introduction

Vector-borne diseases (VBDs), such as malaria, dengue, ZIKA, Chikungunya, and Japanese Encephalitis, impose an important global burden on public health in the past and present. These diseases are not communicable directly among humans, but when favorable conditions are formed for the interaction of pathogens, hosts, and the environment [1]. In recent years, the reproduction and spreading of insect-borne diseases become more widespread with the change in social and other environmental factors such as international trade and global climatic alterations, and the threat to human health from insect-borne diseases is increasing [2]. According to WHO's latest World Malaria Report, there were an estimated 241 million malaria cases and 627 000 malaria deaths worldwide in 2020, which represents about 14 million more cases in 2020 compared to 2019 and 69 000 more deaths. Besides, from September 2019 to November 2021, Dengue was endemic in Pakistan with a total of 102,404 cases including 278 deaths (case fatality ratio (CFR): 0.27%) have been reported. Hence, we need to face the emerging and re-emerging major VBDs and the challenges of their control.

Worryingly, there are currently no effective vaccines or drugs for most VBDs due to the amazing rate of mutation of the virus. Therefore, vector control is the most important means to control VBDs. In 2017, WHO published the global vector control response: an integrated approach for the control of VBDs that mentioned that an estimated 663 million malaria cases were averted in Africa, more than half of which was due to the widespread deployment and measures of vector control. Hence, effective vector control interventions also can dramatically reduce disease treatment costs.

The larvae of vectors are usually targeted with pesticides and other insect growth regulators, which is an available method for controlling many VBDs. Different strategies such as indoor residual spraying and insecticide-impregnated bed nets are also applied. However, the “3R” problems (resistance, residue, and rampant) caused by the applications of these chemical treatments cannot be ignored. Insecticide resistance plays an important role in difficulties in vector control; a variety of vectors such as mosquitoes [3], ticks [4], and lice [5] were found to be resistant to chemical pesticides in different countries and regions. With the development of resistance, the dosage of chemical pesticides continues to increase, and pesticide residues become more and more serious. Researchers found that there were 113 pesticide residues in drinking water samples from 31 countries worldwide [6]. In addition, a study observed a positive exposure-response relationship for 31 pesticides, which concluded an increased risk of cancer among humans [7]. Therefore, alternative interventions with different active ingredients, capable of controlling insecticide-resistant vectors which transmit outdoors, are urgently required to ensure the sustainability of insect control. Nowadays, NPs provide a new option for controlling vectors with the development of nanotechnology. According to Benelli's review, in addition to mosquitoes that transmit encephalitis and Zika, Au NPs can be used against insect vectors that transmit leishmaniasis and trypanosomiasis, such as ticks, flies, and sandflies [8]. Au NPs are not the only kind of nanoparticles effective against insect vectors, but it was found that different kinds of nanoparticles NPs displayed insecticidal activity against vectors, including TiO_2_, Ag, CuO, and Pd, [9–12]. However, how do NPs work on insects? We have limited knowledge about the rationales for their enhanced toxicity at low concentrations. The latest review mentioned that the toxicity of nanoparticles is not followed according to their physical-chemical properties, such as shape, size, surface area, surface charge, solubility, and others. They provided a hypothesis that the number of atoms/ions/molecules per NPs is the source of toxicity [13]. Indeed, this hypothesis needs to be verified. Not only be used as an effective pesticide for insects but NPs can also be added as a new composition for pesticides [14–16]. Cao reported mesoporous silica NPs with a double-shelled hollow structure to deliver pyraclostrobin against the fungus *Phomopsis asparagi* [17]. However, with the deepening of the research, simply loaded drugs can no longer be satisfied the demand of people, and the controlled release nanosized pesticide systems based on NPs came into generation. For example, Shan synthesized a biodegradable and light-responsive amphiphilic polymer, which is stable without UV, and the release rate of pesticide from the NPs gradually increased after treatment with UV [18]. Except for controlled-release drugs, studies showed that NPs can reduce pesticide consumption by protecting active ingredients against hydrolysis and photolysis, which is beneficial to the environment [19–21]. On the other hand, the greener synthesis methods of NPs are more respectful to the environment compared to chemical pesticides. NPs synthesized using biological resources such as plants and plant extracts, bacteria, fungi, yeast, and algae as precursors show low toxicity and high biocompatibility [22–24]. Although previous studies show the potential application of NPs on insects related to public health, the safety of NPs and their influence on enemies remain unknown. Zielinska summarized the nanoecotoxicology of polymeric NPs, showing no risk to the environment or human health in their potential applications [25]. However, the other review revealed the two opposite conclusions. NPs can promote the growth of plants in lower concentrations by promoting photosynthesis and increasing the size of the xylem and phloem. Higher concentrations of NPs can also inhibit the growth of plants by destroying the cellular structure of plants [26]. However, in how to define the high and low concentrations of different nanoparticles, there is no clear standard. In this review, we focus on the application and development of nanoparticles (NPs) for vector control, discussing the lethal mechanism of NPs to vectors and the safety of nanoparticles in the environment, which can explore the prospect of applying nanotechnology in the prevention and control of vectors.

## 2. Classification of Nanoparticles against Insects

We analyzed 425 journal articles which adopted to search the following keywords initially: “nanoparticles against insect,” “NPs against insect,” and “metal nanoparticles against insect,” in PubMed. The thrree major types of nanoparticles (NPs) were identified in this review (Figure 1). Type 1 are metal-based NPs (for example, Ag, Cu, and Ti) which is the most widely used to resist insect, Type 2 are nonmetal-based NPs (for example, Si and Ca), and Type 3 include some complex polymers (for example, chitosan and plant extract). For Type 1 reagents, the element with the largest proportion is Ag, due to its significant impact on insect antioxidant and detoxifying enzymes, leading to ROS-mediated apoptosis, DNA damage, and autophagy [27]. In Type 1, most metals work in this way. However, the main insecticidal principle is different in Type 2; for example, the toxicity of SiO_2_ NPs is due to desiccation, body wall abrasion, and spiracle blockage [28], followed by physical sorption of waxes and lipids, leading to insect dehydration. In addition, nanomaterials used as insecticides can be classified according to different functions. Type 1 mainly includes NPs for directly using as insecticides, and metal-based NPs are the most widely applied in this type. In Type 2, NPs serve as carriers to encapsulate active ingredients to control insects. The first nanoabamectin pesticide recently approved in China adopts the three-dimensional reticulated nanomaterials as the carrier and uses the reticulated nanoscale drug-loading space inherent in the structure of nanomaterials to achieve encapsulation of raw materials without agglomeration (Pesticide Registration Certificate No. PD20210374).

## 3. Different Methods of NPs Synthesis

According to the discipline classification of synthesizing NPs, it can be divided into physical, chemical, and biological methods (Figure 2). The physical method refers to slicing bulk material to get nanosized particles, which mainly includes vacuum condensation, the evaporation-condensation method, and the mechanical ball grinding method [29]. Conversely, the chemical method creates nanostructures by controlling the deposition and growth of atoms and molecules, including solvothermal [30], sol-gel [31], and microemulsion methods [32]. As the most widely used chemical method, the superior advantage of the solvothermal method is the use of no catalysts, but the synthesis mostly prefers toxic solvents to fabricate required materials [33]. However, with the development of synthetic technology, many simpler methods without the use of harsh chemicals to prepare NPs were presented. Li reported a novel solvothermal approach to synthesizing carbon nanoparticles (CNPs), in contrast with previous methods, this synthesis process uses glucose and ammonium oxalate as the carbon source and glycol as the solvent, and neither strong acid treatment nor further surface modification was necessary [34]. The current advancements in solvothermal synthesis methods for NPs indicate that there are many chemical synthesis research opportunities.

Nevertheless, the latest research proposal is the biological method. Nowadays, 1917 articles have been published on PubMed in 2021 (keywords: bio nanoparticle). As an emerging green-synthesis strategy in nanotechnology, the biological method uses living templates that include plants and microorganisms such as plant extracts, viruses, bacteria, and other biomolecules for the synthesis of NPs. Recently, products approach to synthesizing NPs has focused on the use of plant components. These plant-derived nanopesticides can also be subdivided into different types based on their usage, such as plant-derived NPs and nanoemulsions prepared with essential oils extracted from plant parts. For example, iron oxide (Fe_3_O_4_) NPs are synthesized by a *Rhus Coriaria* extract and possess better and enhanced properties than the chemical method [35], and CopaPlu nanoemulsion also showed great antibacterial activity against *Paracoccidioides*. In addition, plants such as *Melia azedarach* leaf, *Azadirachta indica* leaf, and Nasturtium officinale are also explored for the synthesis of Cu-ZnO, CuO, and MoO_3_ NPs [36–38]. In these studies, the presence of phytochemicals in their extract functions as natural stabilizing and reducing agents for NPs production. Furthermore, enzymes and other biomolecules produced by microorganisms can also reduce metal ions to metal NPs. Different microbial such as *Saccaropolyspora hirsute* and *B. licheniformis* are also used in the synthesis of silver, ZnO, and NPs [39, 40]. By the way, the employment of different biological as reducing and stabilizing agents leads to biosynthetic NPs with optical properties, including different sizes, shapes, and differential functional properties on vectors [41, 42]. In a study, different ZnO NP shapes were obtained from *Fusarium keratoplasticum* and *Aspergillus niger*, where *A. niger* synthesized nanorod-shaped NPs showed enhanced antibacterial properties against pathogenic bacteria and UV-protection than *F. keratoplasticum* synthesized hexagonal NPs [43]. Generally speaking, bioderived NPs are regarded as safe, biocompatible, and environmentally friendly particles that cause less harmful effects to human health but are also time-consuming biological screening and expensive. There are pros and cons to different synthesis methods, and the appropriate synthesis method should be selected according to the requirements (Table 1).

## 4. Application of NPs in Vector-Insects

### 4.1. Toxicity of NPs to Insects

The application of NPs obtained through various synthetic pathways as new pesticides has attracted more attention recently. In the last 5 years, more than 600 studies outlining the toxicity of NPs towards various vector-insects have been published. These NPs including gold, silver, titanium oxide, semiconductors, and silica-based nanomaterials have been tested against a wide range of vectors, covering mosquito, lice, and fly [16, 51]. Among all, the large majority of the researchers focused on mosquito vectors due to their huge ecological and physiological plasticity [52]. According to research, most of NPs have obvious acute toxicity against mosquito (Table 2). The published literature was carried out to examine the effectiveness of *Nelumbo nucifera* synthesized Ag NPs against larvae of *An. subpictus* (LC_50_ = 0.69 mg/L) and *Cx. quinquefasciatus* (LC_50_ = 1.10 mg/L) [63]. Palanisamy describes the toxicity of Ag NPs biosynthesized using cheap leaf extract of *Berberis tinctoria* against larval instars (I–IV) of *Ae. Albopictus* with LC_50_ of 4.97 ppm (I instar), 5.97 ppm (II), 7.60 ppm (III), and 9.65 ppm (IV) [64]. Notably, the NPs obtained as described above showed different toxicity against mosquitoes, even if they are the same NPs. Barik tested the three types of silica NPs, including lipophilic, hydrophilic, and hydrophobic, to assess the larvicidal properties of different mosquito species. In *Ae. aegypti*, the LC_50_ was 5-fold less than hydrophilic when treated with hydrophobic silica NPs [65].

Besides, a recent review by Benelli pointed out that NPs could not only be used as mosquito larvicides, ovicides, and adulticides [66, 67] but also reduce mosquito longevity and fecundity [68]. In Thelma's work, the synthesized Ag NPs exhibited significant ovicidal activity. The LC_50_ values for the ovicidal activity were 13.96 ppm, 63.31 ppm, and 24.54 ppm for *Ae. aegypti*, *Cx. quinquefasciatus,* and *An. stephensi,* respectively, which revealed that *Ae. aegypti* was more susceptible to Ag NPs followed by *Cx. quinquefasciatus* and *An. stephensi* [53]. In other studies, growth inhibition was also found in *An. stephensi* and *Cx. quinquefasciatus* at all the concentrations tested in silica NPs [65].

### 4.2. NPs Act as Transport Agents against Vector Insert

Pesticide microencapsulation technology is to encapsulate liquid or solid pesticides in capsule materials to prepare tiny capsule preparations with a particle size of 0.1–10.0 *μ*m, to protect the active ingredients of pesticides from light, air, and other external factors. Decomposition, especially for environmentally sensitive pesticides, making them into microcapsule formulations can greatly improve their effective utilization and achieve high-efficiency mosquito killing effects [69]. In addition, microencapsulation technology not only has the advantages of prolonging drug release time, reducing solvent harm, improving drug efficacy, and improving stability [70] but also can play a huge potential in improving the performance of drug preparations. The technology of microencapsulation enables nanotechnology to work. Compared with traditional drugs, the use of nanomaterials as carriers for drug delivery can protect drugs, delay drug release, improve drug utilization, and reduce drug side effects, so it has more obvious advantages in the biological field (Figure 3).

Some selected nanomaterials, such as ZIF-8, have been tested to stabilize and boost the efficacy of dinotefuran against vector [71]. Zhang adopted a nanocarrier (star polycation, SPc) based on electrostatic interaction with the fluorine group in flufenoxuron to form a flufenoxuron/SPc complex, which reduced the particle size of flufenoxuron from 933 nm to 70 nm and significantly improved larval mortality [72]. Among them, the nanohollow microsphere has an internal cavity structure that can be used to load other small molecule substances, which can efficiently load drugs and proteins to achieve the purpose of targeted delivery. For example, SiO_2_ is classic mesoporous material with outstanding properties such as biocompatibility, pore volume, and specific surface area. Studies confirm that SiO_2_ NPs are relatively stable in water and phosphate-buffered saline, but in cell media, the release of drug molecules can be regulated by controlled corrosion of silica [73]. In addition, NPs have high UV reflectivity and strong stability, which can be used for the protection of light-sensitive drugs. After the *Bacillus thuringiensis,* chitinase was loaded with silica NPs, the pH tolerance, thermal stability, and UV resistance were improved, and the insecticidal activity against *Caenorhabditis elegans* was enhanced [74]. Mesoporous silica also could protect protein Cry 5B from nematode pepsin digestion, while relatively rapidly transporting protein into the intestinal lumen of nematodes [75]. Besides protecting the drug from consumption, the use of NPs could enhance the solubility of insecticides. Water-soluble insecticides can be prepared by modifying chitosan and porous silica-based NPs [76–78]. The use of solid lipid mixtures of NPs can also solve the evaporation or volatilization problems associated with the application of insecticides. All these studies highlight the potential advantages of NPs.

### 4.3. Mode of Action of NPs against Vector Insects

Studies have shown that the insecticidal effect of NPs on vector insects occurs in the following ways:

- Due to the scale effect of NPs, the adhesion of pesticides in the environment can be improved, increasing the possibility of insect exposure to NPs in the environment. After that, NPs could dehydrate cells through stratum corneum adsorption, leading to several morphological and histological abnormalities in insects. Among different NPs, silica and aluminum are represented to bind with the cuticle layer of ticks, leading to physical uptake of lipids and waxes, cell dehydration, and eventual cell death [79] (Figure 4(a)). Experiments by Sultana found that the carbon-dotted silver NPs had high toxicity to *Anopheles stutzeri* and *Culex quinquefasciatus.* SEM analysis in this experiment showed that the above carbon-dotted silver NPs caused deformation of larvae, while X-ray analysis proved nanohybrids in the treated. The presence of Ag in mosquito tissues suggests that their death may be due to the toxicity of nano-Ag at the cellular level. In addition, HR-TEM also showed stratum corneum and cellular tissue damage [80]. Third-instar *Aedes aegypti* larvae exposed to ZnO NPs (1.57 mg/mL, 24 hours) prepared from Lobelia were found to have abdominal contractions, altered thorax shape, midgut lesions, and loss of lateral hairs, anal gills, and brushes, while the accumulation of ZnO NPs was observed in the chest and abdomen [81].
- NPs enter the insect body, causing oxidative stress in the insect, destroying the protein in the insect body, and disturbing the normal physiological function of the insect. *In vivo* studies, DNA damage and oxidative stress have been found when cellular uptake NPs [82]. Previous research studies have shown that NPs have insecticidal activity due to its cytotoxicity. Some NPs, such as TiO_2_, can absorb UV in the environment, the electrons are excited to become highly active after absorbing energy, and holes are generated in the valence band. The oxygen in the air combines with the e− to produce O_2_−. H_2_O undergoes oxidation reaction with produced holes to generate reactive oxygen species (ROS), such as H_2_O_2_, O_2_−, and H_2_O_2_ reacting with glycosides, unsaturated fatty acids, proteins, and other substances in the cell, resulting in the death of cells (Figure 4(b)). Besides, the metal ions contained in the material enter the cell during the process of outward release and bind to the amino acids S and P in proteins, reducing cell membrane permeability [83]. Once inside cells, NPs may cause damage to DNA and inhibit the activity of intracellular enzymes [84]. Very recently, Chimkhan outlined that Ag NPs ingested by *Bacillus thuringiensis* led to mortality and detrimental effects on *Aedes aegypti* larvae. The results showed that six protein expressions in *A. aegypti* larvae were involved in DNA and protein damage, inhibition of cell proliferation, and cell apoptosis, indicating that NPs can affect basic physiological regulation in insects [85].
- The expression of target genes in insects is affected after NPs enter the body of the insect. The effect of NPs on gene expression in insects was published in 2011, and Nair and Choi evaluated the expression of GST genes, which are linked with the occurrence of oxidative stress after *Chironomus riparius* had been exposed to the different concentrations of Cd and Ag NPs for various time [86]. The result shows that all GST genes have up-down regulation to varying levels; among them Delta3, Sigma4, and Epsilonl GST classes have the highest expression levels. However, the expression of genes is not static. Studies have shown that after short-term (24 h) exposure to nanoinsecticides, the expression of detoxification-related genes decreases, but after long-term (48 h) exposure, the expression of detoxification-related genes (*P-gp* and *hr96*) increases significantly. Expression of reproductive system-related genes (*cyp314*, *vtg*, and *dmrt93*) varies with concentration and time [87]. Recently, Zhang analyzed the effect of lufenuron/SPc nanocomplexes on insect gene expression by RNA-seq technology and found that it not only significantly downregulated insect cuticle-related genes (*cut*) and inhibited the formation of insect cuticles but also upregulated endocytosis-related genes, promoting drug intake [72]. This suggests that NPs can improve insect toxicity by affecting insect gene expression (Figure 4(c)).

### 4.4. The Safety of the NPs

The small size, large surface, and more active area account for the extensive use of NPs in various applications, such as in drug delivery [88], diagnostics [89], food science [90], electronics [91], and several other biological and nonbiological areas. With the increased interest in nanotechnology in the last decade, the safety of NPs in the environment has also been considered. Therefore, in addition to the toxicity of NPs to vector insects, the impact of NPs on nontarget organisms in the environment has become the focus of attention. In a study, Chakraborty et al. used zebrafish as a model organism to investigate the toxic effects of silver NPs, gold NPs, and several metal oxide NPs (TiO_2_, Al_2_O_3_, CuO, NiO, and ZnO) on it [92]. The correlation between successful hatching efficiency and embryotoxicity is an important parameter for evaluating nanotoxicity. The researchers learned about embryotoxicity by assessing the relationship between hatching success and hours after exposure to TiO_2_ NPs. The study found that titanium dioxide NPs can cause premature hatching of zebrafish embryos in a dose-dependent manner. Through gene ontology (GO) and Kyoto Encyclopedia of Genes and Genomes (KEGG) enrichment analyses, Lu et al. found that silver NPs caused the accumulation of reactive oxygen species (ROS) and malondialdehyde (MDA) in zebrafish embryos, inhibiting the superoxide dismutase (SOD), catalase (CAT), and mitochondrial complex I-V activity, and downregulated the expression of SOD, CAT, and mitochondrial complex I-IV chain-related genes, ultimately leading to zebrafish embryotoxicity [93]. However, some studies have also shown that TiO_2_ NPs can reduce the toxicity of pesticides to zebrafish. To study the bioconcentration and cardiotoxicity mechanism of azoxystrobin (AZ) under the action of TiO_2_ NPs, zebrafish embryos were exposed for 72 h after fertilization. The results showed that the presence of TiO_2_ significantly reduced AZ accumulation in larvae compared with AZ alone and thus notably decreased AZ-induced cardiotoxicity, including changes in gene expression of heart rate, pericardium edema, venous thrombosis, sinus venosus, and bulbus arteriosus distance [94]. This suggests that insecticides mixed with NPs help to slow the release of active molecules, thereby helping to reduce the toxic effects of insecticides [95, 96]. The effects of Ag NPs synthesized by *T. asiatica* aqueous extract on the predation rate of *Culex quinquefasciatus* by zebrafish were also evaluated in indoor and field experiments. It was found that the predation of mosquito larvae was slightly higher than in normal laboratory conditions in the silver-exposed environment, indicating that Ag NPs can be used at low doses to reduce the number of mosquito vectors without adversely affecting the predation of natural enemies [97]. In addition to acute toxicity, whether NPs have long-term toxicity to organisms has also been investigated. Al_2_O_3_ NPs and ZnO NPs are fed uninterrupted daily to rats for 75 days, and the result found that NPs caused hepato-renal toxicity at all parameter levels and inhibited the expression of mitochondrial transcription factor A gene and peroxisome proliferator-activated receptor gamma coactivator [98]. Chronic exposure of the Northern Pike (*Esox lucius*) and their primary prey species Yellow Perch (*Perca flavescens*) to Ag NPs caused the length- and weight-at-age (indices of growth rate) of the Northern Pike decline and the per capita availability of Yellow Perch declined by over 30% [99]. Despite considerable efforts to understand the toxicity and safety of these NPs, many of these questions are not yet fully answered. The differences in the toxicity of these NPs may depend on their biophysical properties, including size, surface area, surface charge, and aggregation state, which have been shown to influence the distribution and deposition of NPs in different organ systems and alter their molecular interactions with various proteins and other macromolecules [100].

### 4.5. Challenges and Opportunities

Nanotechnology is an ecological branch of vector control, and previous studies indicated its great potential for a practical application already, but several questions remain to be solved as follows:

- How to improve the economic efficiency of NPs biosynthesis.
- The potential connection between loading efficiency and the relevant property of NPs, such as size, shape, and crystal structure.
- The mechanism and correlation between the dose of different kinds of NPs and acute or long-term toxicity of organisms.
- Effects of NPs residue on generations of vectors and nontarget organisms in the environment.

The above challenges cannot be solved by short-term experiments, and people should work for long-term experimental results to confirm conclusions.

## 5. Conclusions

Historically and currently, vector control is a very effective means of preventing and controlling infectious diseases. However, environmental changes, pesticide resistance, and population growth have created a new set of challenges for current vector control. There is an urgent need to develop new vector control tools using all our existing interventions, including insecticide and nonpesticide-based control methods. As a rapidly developing new discipline, the application of nanotechnology has been involved in many fields such as medicine, agriculture, catalysis, and biosensing. Compared with traditional chemical and physical methods to synthesize nanomaterials, green synthesis methods have better sustainability and environmental safety. In addition to possibly having some anti-insect effects on their own, NPs can also be effective in carrying pesticides [76–78]. In this review, we found that almost every type of NPs have been used for insect resistance, including metal, nonmetal, and other substances with particle sizes on the nanometer scale. The novel method for obtaining these NPs is the biological synthesis approach, which has better sustainability and environmental safety compared with traditional chemical methods. In addition to possibly possessing insecticidal efficiency on their own, NPs that are synthesized by different methods can also be effective in carrying pesticides, solving the evaporation or volatilization issues associated with pesticide application, and helping to slow the release of the active ingredient, thereby reducing the pesticide's toxic effects. Overall, NPs have provided new ideas for the prevention and control of infectious disease vector insects by elaborating on the insecticide mechanism and safety. Due to the diversity of species, nanoparticles have an immeasurable potential for vector control. Nevertheless, despite efforts to elucidate the mechanisms of nanoparticle toxicity in the three different aspects, our knowledge in the related field is still lacking, the information on the effects of NPs on different types of vector insects is unclear, and the impact of the size, shape, and charge of NPs on various potential mechanisms of action is also to be verified. Because of the uncertainty of the toxicity mechanism of NPs, their sublethal effects on nontarget organisms also require further monitoring, especially genotoxicity and fine physiological and behavioral modifications. In addition, exploring the stability of NPs in the environment, finding suitable standard production methods, and developing commercial products based on nano pesticides are also the keys to the next step to applying NPs in practice.

## Figures and Tables

**Figure 1:** Classification of NPs against insects. NPs used to resist insects can be roughly divided into the three categories according to different properties. Among them, metal-based NPs account for the highest proportion, reaching 63.29%, and nonmetal-based NPs, such as Si- and C-based, account for only 14.35%.

**Figure 2:** The three different synthesis methods of nanoparticles: the chemical method: different substances react chemically to form nanoparticles, the physical method: the particle size of the material is made to the nanometer scale by physical means, and the biological method: synthesis of nanoparticles from biological extracts.

**Figure 3:** Nanoparticles act as carriers to loading pesticides. Nanoparticles encapsulate pesticides to protect them from external factors. Meanwhile, under the stimulation of these external factors, active components will be released to achieve the controllable effect.

**Figure 4:** Mode of action of NPs against vector insects. (a) The NPs bind to the body surface of vectors, leading to the physical absorption of lipids and waxes, causing cell dehydration and deformation of the larvae. (b) Photocatalytic mechanism of titanium dioxide, generating peroxides such as reactive oxygen species causing oxidative stress in vectors. (c) Several ways in which NPs can cause the death of vectors by affecting cells: (1) metal NPs release metal ions that reduce the permeability of cell membranes and cause cytoplasmic leakage; (2) NPs reduce enzyme activity; and (3) NPs cause DNA damage and also affect the related gene expression.

**Table 1:** Advantages and disadvantages of different synthesis methods.

	Advantages	Disadvantages
Physical methods	Simple methodology [44]	The lower yield of NPs
		Higher energy-consuming
		Higher input cost [45]

Chemical methods	Homogenous NPs with high accuracy	The usage of toxic chemicals [46, 47]
	The consumption of less energy [48]	

Biological methods	Do not involve toxic chemicals in the preparation protocols	Highly demanding
		Time-consuming
		Requiring technology and practical microbiological experience to ensure cell culture and nanoparticle purification under aseptic conditions [49, 50]

**Table 2:** Various NPs with their applicative measures against the different mosquito species.

Nanoparticles	Source	Target's species	Lethal indices (LC_50_)
Ag	*Bacillus marisflavi* [53]	*Ae. aegypti*	13.96 ppm
Ag		*Cx. quinquefasciatus*	24.54 ppm
Ag		*An. stephensi*	29.14 ppm

Ag	*Ipomoea batatas* [54]	*Ae. aegypti*	17.578 *μ*g/mL
Ag		*Cx. quinquefasciatus*	10.069 *μ*g/mL
Ag		*An. stephensi*	12.568 *μ*g/mL

Ag	*Cassia roxburghii* [55]	*Ae. aegypti*	26.35 *μ*g/mL
Ag		*Cx. quinquefasciatus*	28.67 *μ*g/mL
Ag		*An. stephensi*	31.27 *μ*g/mL

Au	*Parmelia sulcata* [56]	*Ae. aegypti*	70.16 ppm

ZnO	*Cucurbita* [57]	*Cx. tritaeniorhynchus*	39.007 ppm

ZnO	Chemical method [58]	*Cx. quinquefasciatus*	291.0 mg/L

ZnO	*Pseudomonas aeruginosa* [59]	*Culex pipiens*	75 ppm

ZnO	*Cucurbita* [59]	*Cx. tritaeniorhynchus*	44.68 ppm

MgO	*Penicillium chrysogenum* [60]	*An. stephensi*	12.5–15.5 ppm

MgO	Chemical method [58]	*Cx. quinquefasciatus*	83.4 mg/L

CuO	Chemical method [58]	*Cx. quinquefasciatus*	100.8 mg/L

CuO	*Tridax procumbens* [61]	*Ae. aegypti*	4.209 mg/L

SiO_2_	Chemical method [58]	*Cx. quinquefasciatus*	27.81 mg/L

Se	*Nilgirianthus ciliatus* [62]	*Ae. aegypti*	0.92 mg/L
